# Pharmacological Study on Total Glycosides of Xiebai Protecting against Depression Model

**DOI:** 10.1155/2022/5498130

**Published:** 2022-03-29

**Authors:** Hui Zhao, Meiqiong Jiang, Mingsan Miao

**Affiliations:** ^1^Department of Pharmacology, School of Pharmacy, Chengdu University of Traditional Chinese Medicine, Chengdu 611137, China; ^2^College of Postgraduates, Henan University of Chinese Medicine, Zhengzhou 450000, China

## Abstract

**Objective:**

To observe the effect of total glycosides of Xiebai on chronic unpredictable stimuli in rats. Changes of serotonin (5-HT), dopamine (DA), norepinephrine (NE), serum corticosterone (CORT), adrenocorticotropic hormone (ACTH), organ index, and histopathology in brain tissue, to explore the treatment and characteristics of total white glucosides in depression model, were prepared by different stimuli in 21 days.

**Methods:**

Depression models were replicated by 21 days of chronic mild stimulation in rats. Finally, the levels of CORT and ACTH in the serum of rats with depression model and the levels of NE, DA, and 5-HT in brain homogenates were determined. The thymus and spleen wet weight of each group were measured, and the organ index was calculated. The thymus and pituitary were observed under the light microscope. Pathological changes of the hypothalamus, adrenal gland, and spleen and behavioral indexes of rats in each group were determined.

**Results:**

The results of the experiment showed that 21 days of chronic unpredictable stimulation significantly improved the behavioral response of the model group, and the levels of corticosterone and adrenocorticotropic hormone in the serum and the indicators in the brain homogenate significantly changed, affecting the relevant tissues. The index changes and the results of the combination can prove that this modeling method can be used for the preparation of depression models. The total white glucoside group can significantly improve the above effects, demonstrating that total glucosides of glucoside have a good therapeutic effect on the rat model of depression.

**Conclusion:**

The chronic unpredictability of the total dose of Xiebai glycosides can significantly improve the levels of NE and DA and the levels of serum CORT and ACTH in the brain homogenate of depressive model rats and improve the immune function of the body.

## 1. Introduction

The main symptoms of depression are loss of pleasure and lack of interest [1]. The clinical symptoms are divided into three categories: core symptoms, psychological symptoms, and physical symptoms. With the change of lifestyle, the incidence of depression is also increasing year by year [2]. Recently, studies have found that the occurrence of depression is accompanied by the emergence of digestive diseases, cancer, etc., thus increasing the difficulty of treatment of this disease [3]. Western medicine believes that depression is a psychiatric disease. The cause of disease is caused by excessive activity of central nervous system excitatory transmitters or excessive activity of inhibitory transmitters. Therefore, the therapeutic effect of Western medicine in the treatment of depression to selectively activate excitatory transmitters is passed. The reuptake of excitatory addresses is blocked by nerve endings to increase excitatory transmitter levels [4]. From the perspective of Chinese medicine, depression is not a single pathological disease and can be divided into various types according to its characteristics and pathogenesis [5]. Depression is mainly caused by damage to the liver, heart, and spleen and dysregulation of blood and blood. Clinically, the combination of false and real, the beginning of the disease is due to the damage of visceral blood and yin and yang, and is more common [6]. Hepatic dysfunction is abnormal; spleen transporting water valley is unfavorable; abnormal liver function, poor spleen transport of water and valley, impaired heart function, disorders of viscera, yin and yang, qi, and blood are the pathogenesis of depression [7]. Xiebai has the effect of clearing the yang and stagnation of the qi and is used clinically for the treatment of chest pain, heartache, fullness and pain, diarrhea, and other diseases [8]. Modern research suggests that Xiebai has the effect of alleviating the symptoms of depression. Clinically, there are reports of using Xiebai prescription to treat depression [9]. Therefore, this study used Chinese medicine Xiebai to study the Xiebai total glycosides in Xiebai. The effects of a depressed rat model are shown in Figure 1.

## 2. Experimental Material

### 2.1. Experimental Animals

Wistar male rats, 180–220 g, SPF grade, were provided by Shandong Lukang Pharmaceutical Co., Ltd. (certificate no. 0017183; laboratory certificate no. SYXK (Yu) 2010-001; ethical batch no. DWLL15010017). Approval was obtained from Animal Experimental Ethics Committee of Henan College of Traditional Chinese Medicine, approval time: September 20, 2013.

### 2.2. Experimental Drugs

Xiebai total glycosides, Xiebai was pulverized into a coarse powder, and added with 10 times of 70% ethanol under reflux for 2 times, each time 1.5 h; the two alcohol extracts were combined, concentrated under reduced pressure to an alcohol-free taste, and dispersed with distilled water (concentration of 0.2 g of medicinal material/ml) as a sample solution. After D101 resin, flow sample, let stand for 5 hours to be fully adsorbed, first wash with 5 times column volume of distilled water, discard the water solution, and then remove the impurities by 5 times column volume 10% ethanol, and finally use 6. The column volume was eluted with 70% ethanol, the eluate was collected and evaporated to obtain a powder, and the content was determined to be 52.3%. Fluoxetine hydrochloride, Changzhou Four Medicine Co., Ltd., product batch number: 20121023.

### 2.3. Experimental Reagents

The following experimental reagents were used: sodium carboxymethyl cellulose, Tianjin Hengxing Chemical Reagent Manufacturing Co., Ltd., batch number: 20110728; glucose injection, Kaifeng Pharmaceutical (Group) Co., Ltd., batch number: 13080501; rat 5-HT ELISA test kit, R&D, batch number: 20131101B; rat DA ELISA test kit, R&D company, batch number: 20131101B; rat NE ELISA test kit, R&D company, batch number: 20131101B; rat CORT ELISA test kit, R&D company, batch number: 20131101B; and mouse ACTH ELISA test kit, R&D, batch number: 20131101B.

### 2.4. Experimental Instruments

The following experimental instruments were used: high-speed refrigerated centrifuge, produced by Zhongjia Branch of HKUST Innovation Co., Ltd., model KDC-160HR; adjustable pipette, Shanghai Leibo Analytical Instrument Co., Ltd.; and microplate reader, produced by American BIO-RAD, model 680.

## 3. Experimental Methods

### 3.1. Modeling and Administration

Sixty male Wistar rats weighing 180–220 g were divided into 6 groups: blank group; positive group; model group; and groups with small, medium, and large doses of Xiebai total glycosides. Rats in the blank group were not given any stimulation, and single-cage monoculture was not performed. The rats in the model group and the administration group were single-cage single-culture [10].

The rats in the depression group received 21 days of chronic mild unpredictable stress stimulation, and the simulation method was divided into 7 types as follows [11]. The first type is ice water swimming. The rats were placed in a container filled with cold water at 4°C for 5 minutes. During the process, the rat's foot just touched the bottom end of the container and was taken out after stimulation. The second type is heat stress. The oven was adjusted to 45°C. Constantly, the rats were placed in it for five minutes and then taken out. The third type is free access to water for 24 h. The fourth type is fasting for 24 h. The fifth type is clip tail. The rat was fixed, the tail was exposed, and the hemostasis was clamped 1 cm from the base of the tail. The force should not be too large; the rat can scream; after 1 min stimulation, release it. The sixth type is wet padding (200 ml water per 100 g pad). The seventh type is overnight illumination for 24 h. The above-mentioned stimuli were randomly arranged during the 21-day modeling process, and one stimulation method was used per day. Each stimulation was not repeated more than three times, to avoid the adaptability of the rats.

Method of administration is as follows: This experiment was carried out utilizing modeling while administering. The positive group was intragastrically administered with fluoxetine hydrochloride suspension 6.6 mg kg^−1^. The groups with small, medium, and large doses of total white glycosides were intragastrically administered 50 mg kg^−1^, 100 mg kg^−1^, and 200 mg kg^−1^, respectively. The blank group and the model group were given the same volume of distilled water and were intragastrically administered once a day for 21 days.

### 3.2. Observation Items and Detection Methods

The [12–14] sucrose consumption test was performed on each group of rats for 20 days, and the swimming time was measured at 21 days after administration. One hour after the last administration, humane and ethical blood collection was carried out, and the serum was separated for the determination of CORT and ACTH. Then, the rats were sacrificed by cervical vertebrae, the thymus and spleen were taken, the blood on the organs was blotted with filter paper, and the weight was calculated. The index of each organ (the ratio of organ weight (mg)/body weight (g)) was calculated. After taking brain tissue homogenate, the levels of DA, NE, and 5-HT in brain tissue were measured, and the hypothalamus and pituitary were simultaneously separated. Thymus, spleen, adrenal gland, and brain tissue were fixed in 10% formaldehyde solution, embedded in paraffin, sectioned, and HE-stained, and histomorphological changes were observed under the light microscope.

#### 3.2.1. Sugar Consumption Test

On the 21st day of the experiment, fast water was added to the kettle containing 1% sucrose, and the sugar consumption of the animals within 24 hours was calculated.

#### 3.2.2. Forced Swimming Test

On the 21st day of the experiment, after adding an appropriate amount of water to the animals, each animal was placed in a limited environment with an appropriate amount of water, so that it struggled but could not escape, and the record was in the environment. The animals produce parameters in the process of a desperate state.

#### 3.2.3. Kit Detection Method

The eyeballs were removed and coagulated at room temperature, serum was separated after centrifugation, and serum corticosterone (CORT) and adrenocorticotropic hormone (ACTH) levels were measured by enzyme immunoassay. After the behavioral test, the levels of monoamine neurotransmitters 5-HT, DA, and NE in brain homogenate were determined by the enzyme-free method.

### 3.3. Statistical Processing Methods

Data analysis uses SPSS 17.0 medical statistical package for statistical processing of data, measurement data is expressed by mean ± standard deviation ($\bar{x}$ ± *s*), and one-way analysis of variance was used for comparison between groups. The LSD method was used for the variance test, the Games–Howell method was used for the variance, and the Ridit test was used for the grade data.

## 4. Results

### 4.1. Effects on Body Weight of Chronic Depression Model Rats

The test results of the weight of each group of rats in the experiment are shown in Table 1.

It can be seen from Table 1 that on the 14th day and the 21st day of stress treatment, the body weight of the model group was significantly lower than that of the blank control group; compared with the body weight of the model group and the positive drug fluoxetine hydrochloride group, the body weight of rats in the large- and medium-dose Xiebai total glycosides group increased significantly (*P* < 0.05, *P* < 0.01).

### 4.2. Effects of Sucrose Consumption and Swimming Time on Chronic Depression Model Rats

The test results of sugar water consumption and swimming time in each group of rats are shown in Table 2.

It can be seen from Table 2 that compared with the blank group, the preference of the model group for syrup is significantly reduced, which proves that the modeling method is feasible; compared with the model group, the positive drug fluoxetine hydrochloride group, large, medium The preference for syrup was significantly increased in the dose of Xiebai total glycosides (*P* < 0.05, *P* < 0.01). Compared with the blank group, the swimming time of the model group was significantly increased (*P* < 0.01), reflecting the increased despair of the unfavorable environment in the depression model rats, suggesting that the modeling was successful. Compared with the model group, the positive drug fluoxetine hydrochloride group and high-dose Xiebai total glycosides group could significantly reduce the time of forced swimming in rats (*P* < 0.05, *P* < 0.01).

### 4.3. Effects of Monoamine Neurotransmitters on Brain Tissue in Rats with Chronic Depression

The contents of 5-HT, DA, and NE in the brain tissue of each group are shown in Table 3.

It can be seen from Table 3 that the levels of 5-HT, DA, and NE in the brain homogenate of the model group were significantly lower than those in the blank group (*P* < 0.01), indicating that the rat model of chronic stress depression was successful. Compared with the model group, the hifalutin hydrochloride group and groups with large, medium, and small doses of Xiebai total glycosides can significantly increase the levels of 5-HT, DA, and NE in brain homogenate (*P* < 0.05, *P* < 0.01).

### 4.4. Effects of Serum ACTH and CORT Levels on Chronic Depression Model Rats

The contents of ACTH and CORT in the serum of each group are shown in Tables 4 and 5.

It can be seen from Table 4 that compared with the blank group, the levels of ACTH and CORT in the serum of the model group were significantly increased (*P* < 0.01), indicating that the rat model of chronic stress depression was successful. Compared with the model group, the fluoxetine hydrochloride group and the groups with large, medium, and small doses of Xiebai total glycosides can reduce the levels of ACTH and CORT in serum (*P* < 0.05, *P* < 0.01).

### 4.5. Effect of Organ Index on Chronic Depression Model Rats

The thymus and spleen index of each group are shown in Table 5.

As can be seen from Table 5, compared with the blank group, the thymus and spleen index of the model group were significantly decreased (*P* < 0.01), indicating that the thymus and spleen atrophy appeared in the rat model of chronic depression and depression. Compared with the model group, the total, small and medium doses of Xiebai hydrochloride in the fluoxetine hydrochloride group can significantly increase the thymus index of the model animals (*P* < 0.01); the fluoxetine hydrochloride group, the large, medium and small doses of Xiebai total glycosides can be The spleen index of the model animals was significantly increased (*P* < 0.05).

### 4.6. Effects of Organ Morphology on Chronic Depression Model Rats

#### 4.6.1. Effect of Hypothalamic Tissue Morphology on Chronic Depression Model Rats

According to the different degrees of changes in the structure, cytoplasm, and nucleus of the hypothalamus in the experimental groups, the pathological histomorphology was divided into four levels using semiquantitative criteria. The rats in each group were tested. The results are shown in Table 6.

According to the Ridit test, it can be seen from Table 6 that compared with the blank group, significant hypothalamic lesions appeared in the model group (*P* < 0.01). Compared with the model group, each drug group can significantly improve the pathological changes of the rat hypothalamus (*P* < 0.01).

#### 4.6.2. Effect on Pituitary Morphology of Chronic Depression Model Rats

In the pituitary tissue of rats, the pituitary gland associated with secretion was mainly observed, and the number of glandular cells falling within 5000 square micrometers of the micro-rectangular area was observed under a high power field (×400 times). The observation results are shown in Table 7.

As can be seen from Table 7, compared with the blank group, the number of gland cells in the model group was significantly different (*P* < 0.01), indicating that the gland cells of the chronic depression rat model were large in volume, active in function, and strong in secretory ability. Compared with the model group, the fluoxetine hydrochloride and the medium dose of Xiebai total glycoside significantly increased the number of gland cells in the model animals (*P* < 0.01).

#### 4.6.3. Effect of Thymus Tissue Morphology on Chronic Depression Model Rats

The thickness of the thymus cortex was measured with a micrometer under the field of light microscopy (×200 times), and the number of lymphocytes pressed against the micrometer was calculated. The measurement results are shown in Table 8.

From Table 8, it can be seen that the number of thymic cortex lymphocytes in the model group was significantly lower than that in the blank group (*P* < 0.01), indicating that the thymus volume was atrophied after the chronic depression model was established in rats. Compared with the model group, the number of cortical lymphocytes was significantly increased in each drug-administered group (*P* < 0.01), and the effect of the large- and medium-dose Xiebai total glycosides group was the best.

#### 4.6.4. Effect on the Morphology of the Adrenal Cortex in Chronic Depression Model Rats

The thickness of the adrenal cortical band and the reticular band was measured with a micrometer under the field of view of the light microscope (×200 times). The measurement results are shown in Table 9.

From Table 9, it can be seen that the thickness of the adrenal cortex in the model group was significantly increased compared with the blank group (*P* < 0.01), indicating that the adrenal hyperfunction was induced in the model of chronic depression in rats. Compared with the model group, the administration group significantly reduced the adrenal cortex thickness (*P* < 0.01), and the optimal effect was obtained with the large dose of Xiebai total glycosides.

#### 4.6.5. Effect of Spleen Tissue Morphology on Chronic Depression Model Rats

The diameter of the spleen germinal center was measured with a micrometer under the field of light microscopy (×200 times). The measurement results are shown in Table 10.

As can be seen from Table 10, compared with the blank group, the diameter of the splenomegaly germinal center of the model group was significantly decreased (*P* < 0.01), indicating that the spleen function decreased after the chronic depression model was established in rats. Compared with the model group, the diameter of the splenomegaly germinal center was significantly increased in each drug-administered group (*P* < 0.01), and the effect of the large- and medium-dose Xiebai total glycosides group was the best.

## 5. Discussion

Depression is a long-term manifestation of a mental illness with a low mood [15]. The clinical manifestations are mostly being unhappy, and severe cases may have grief or even a stiff state [16]. At present, there are many studies on the etiology and pathogenesis of depression [17], mainly including monoamine neurotransmitter deficiency hypothesis and hypothalamic-pituitary-adrenal (HPA) axis negative feedback disorder hypothesis. So, the experiment started with the study of the hypothalamic-pituitary-adrenal axis, to study the regulatory effect of drugs on monoamine neurotransmitters [18].

From the perspective of Western medicine, the incidence of depression involves multiple systems in the body, neurological, endocrine, and immune systems [19]. Chinese medicine believes that depression is often based on the treatment of the liver, spleen, and kidney and adjusting its standard [20]. Shugan Jieyu, clearing fire and removing phlegm, and nourishing the heart and spleen are important treatment rules [21]. Traditional Chinese medicine often uses the method of relieving, regulating qi, activating blood circulation, and relieving depression to relieve and treat depression [22]. Commonly used treatment methods include classification therapy, acupuncture therapy, massage therapy, health guidance intervention, and psychosomatic therapy [23]. Traditional Chinese medicine has rich clinical experience and theoretical foundation behind it in the treatment of depression, but there are also drawbacks such as lack of research, lack of science, and poor regularity of medication [24].

Various active ingredients such as volatile oil and saponin have been isolated from Xiebai [25], including polysaccharides and various essential trace elements, garlic sugar, and glycosides [26]. Modern pharmacological research found that Xiebai has a variety of pharmacological effects such as antidepression-like activity [27], scavenging oxygen free radicals, antioxidation, anti-inflammatory activity, and antibacterial activity [28–33].

By preparing a rat depression model, it was found that Xiebai total glycosides can improve mental activity, reduce the degree of despair, and shorten the desperate time; by affecting the transmission of monoamine neurotransmitters, the neurotransmitters in brain tissue can be significantly increased. Correcting the deficiency of monoamine neurotransmitters (5-HT, DA, and NE content) can regulate the activation of hypothalamic-pituitary-adrenal cortex (HPA) axis function and improve the morphology and function of hypothalamic nerve cells, and inhibition of gonadal function. The secretion of pituitary gland significantly reduces the levels of hormones ACTH and CORT in the serum, enhances the body's immune function, restores the atrophy of the thymus and spleen immune organs, and increases the number of lymphocytes. The experimental results show that Xiebai total glycosides have broad application prospects in the treatment of depression.

## Figures and Tables

**Figure 1:** Technical route of Xiebai intervention model of depression.

**Table 1:** Effect of total glucosides of Xiebai on body weight of chronic depression model rats ($\bar{x}$ ± *s*).

Group	Number of animals	Dose/mg·kg^−1^	1 d	7 d	14 d	21 d
Blank group	10	—	198.1 ± 7.3	250.1 ± 16.8	281.6 ± 9.8^*∗∗*^	300.7 ± 8.7^*∗∗*^
Model group	10	—	195.8 ± 8.0	248.4 ± 15.1	259.7 ± 16.9	269.6 ± 17.0
Fluoxetine hydrochloride group	10	6.6	197.7 ± 8.9	250.1 ± 13.5	280.0 ± 16.6^*∗∗*^	290.5 ± 17.3^*∗∗*^
High-dose Xiebai total glycosides group	10	200	193.5 ± 6.9	239.8 ± 12.3	278.6 ± 12.8^*∗∗*^	292.5 ± 12.8^*∗∗*^
Medium-dose Xiebai total glycosides group	10	100	196.6 ± 8.6	245.1 ± 14.4	272.8 ± 11.3^*∗*^	283.7 ± 11.4^*∗*^
Low-dose Xiebai total glycosides group	10	50	192.5 ± 7.4	248.6 ± 17.9	263.7 ± 11.3	281.0 ± 12.1^*∗*^

*Note*. Compared with the model group, ^*∗*^*p* < 0.05 and ^*∗∗*^*p* < 0.01.

**Table 2:** Effect of total glucosides of Xiebai on syrup consumption and swimming time in rats with chronic stress depression ($\bar{x}$ ± *s*).

Group	Number of animals	Dose (mg·kg^−1^)	Sugar consumption (ml)	Static time (s)
Blank group	10	—	76.9 ± 8.5^*∗∗*^	62.4 ± 12.2^*∗∗*^
Model group	10	—	53.6 ± 7.8	117.1 ± 19.9
Fluoxetine hydrochloride group	10	6.6	67.2 ± 7.6^*∗∗*^	82.7 ± 12.1^*∗∗*^
High-dose Xiebai total glycosides group	10	200	66.9 ± 7.3^*∗∗*^	89.7 ± 16.7^*∗∗*^
Medium-dose Xiebai total glycosides group	10	100	62.0 ± 4.9^*∗∗*^	103.0 ± 16.7^*∗*^
Low-dose Xiebai total glycosides group	10	50	59.9 ± 5.1^*∗*^	107.6 ± 13.5

*Note*. Compared with the model group, ^*∗*^*p* < 0.05 and ^*∗∗*^*p* < 0.01.

**Table 3:** Effect of total glucosides of Xiebai on 5-HT content in chronic stress depression rats ($\bar{x}$ ± *s*).

Group	Number of animals	Dose (mg·kg^−1^)	5-HT (ng·ml^−1^)	DA (pg·ml^−1^)	NE (ng·ml^−1^)
Blank group	10	—	81.12 ± 5.96^*∗∗*^	251.24 ± 17.26^*∗∗*^	85.62 ± 4.91^*∗∗*^
Model group	10	—	58.17 ± 8.62	183.71 ± 17.51	54.42 ± 10.12
Fluoxetine hydrochloride group	10	6.6	73.17 ± 8.21^*∗∗*^	220.32 ± 25.29^*∗∗*^	75.20 ± 12.67^*∗∗*^
High-dose Xiebai total glycosides group	10	200	72.52 ± 11.77^*∗∗*^	210.53 ± 24.42^*∗∗*^	69.93 ± 14.17^*∗∗*^
Medium-dose Xiebai total glycosides group	10	100	72.76 ± 12.28^*∗∗*^	214.50 ± 15.74^*∗∗*^	68.32 ± 10.18^*∗∗*^
Low-dose Xiebai total glycosides group	10	50	67.97 ± 7.33^*∗*^	203.63 ± 19.84^*∗*^	66.22 ± 10.92^*∗*^

*Note*. Compared with the model group, ^*∗*^*p* < 0.05 and ^*∗∗*^*p* < 0.01.

**Table 4:** Effect of total glucosides of Xiebai on ACTH content in chronic stress depression rats ($\bar{x}$ ± *s*).

Group	Number of animals	Dose (mg·kg^−1^)	ACTH (pg·ml^−1^)	CORT (ng·ml^−1^)
Blank group	10	—	26.68 ± 4.26^*∗∗*^	126.19 ± 32.73^*∗∗*^
Model group	10	—	34.70 ± 3.46	191.58 ± 27.65
Fluoxetine hydrochloride group	10	6.6	25.99 ± 5.70^*∗∗*^	147.34 ± 31.75^*∗∗*^
High-dose Xiebai total glycosides group	10	200	30.75 ± 2.68^*∗*^	141.30 ± 28.32^*∗∗*^
Medium-dose Xiebai total glycosides group	10	100	31.59 ± 2.17^*∗*^	156.11 ± 29.79^*∗*^
Low-dose Xiebai total glycosides group	10	50	35.05 ± 3.72	167.62 ± 31.96^*∗*^

*Note*. Compared with the model group, ^*∗*^*p* < 0.05 and ^*∗∗*^*p* < 0.01.

**Table 5:** Effect of total glucosides of Xiebai on spleen index in the thymus of rats with chronic stress depression ($\bar{x}$ ± *s*).

Group	Number of animals	Dose (mg·kg^−1^)	Thymus index (mg·g^−1^)	Spleen index (mg·g^−1^)
Blank group	10	—	1.725 ± 0.513^*∗∗*^	3.019 ± 0.531^*∗∗*^
Model group	10	—	1.212 ± 0.323	2.389 ± 0.211
Fluoxetine hydrochloride group	10	6.6	1.880 ± 0.433^*∗∗*^	2.843 ± 0.570^*∗*^
High-dose Xiebai total glycosides group	10	200	1.953 ± 0.407^*∗∗*^	2.868 ± 0.454^*∗*^
Medium-dose Xiebai total glycosides group	10	100	1.904 ± 0.334^*∗∗*^	2.857 ± 0.364^*∗*^
Low-dose Xiebai total glycosides group	10	50	1.761 ± 0.396^*∗∗*^	2.791 ± 0.335^*∗*^

*Note*. Compared with the model group, ^*∗*^*p* < 0.05 and ^*∗∗*^*p* < 0.01.

**Table 6:** Effect of total glucosides of Xiebai on pathological changes of the hypothalamus in chronic depression model rats.

Group	Number of animals	Dose (mg·kg^−1^)	—	+	++	+++	*P*
Blank group	10	—	10	0	0	0	<0.01
Model group	10	—	0	0	2	8	
Fluoxetine hydrochloride group	10	6.6	3	6	1	0	<0.01
High-dose Xiebai total glycosides group	10	200	7	2	1	0	<0.01
Medium-dose Xiebai total glycosides group	10	100	2	7	1	0	<0.01
Low-dose Xiebai total glycosides group	10	50	1	7	2	0	<0.01

*Note.* “—”: nerve cells have a clear structure and no abnormality; “+”: nerve cells shrink in size, and cytoplasm is less; “++”: nerve cells shrink in size, the cytoplasm is less, and cytoplasmic Nissl bodies disappear; “+++”: nerve cells are reduced in size, with less cytoplasm and pyknosis, or have a neurotic phenomenon.

**Table 7:** Effect of total glucosides of Xiebai on pituitary pathological changes onchronic depression model rats.

Group	Number of animals	Dose (mg·kg^−1^)	Number of cells
Blank group	10	—	47.2 ± 2.2^*∗∗*^
Model group	10	—	38.2 ± 2.1
Fluoxetine hydrochloride group	10	6.6	41.6 ± 2.8^*∗∗*^
High-dose Xiebai total glycosides group	10	200	46.3 ± 1.6^*∗∗*^
Medium-dose Xiebai total glycosides group	10	100	44.3 ± 1.3^*∗∗*^
Low-dose Xiebai total glycosides group	10	50	40.1 ± 1.6^*∗*^

*Note*. The number of cells that fall within the frame is small, indicating that the gland cells are large and active. Compared with the model group, ^*∗*^*p* < 0.05 and ^*∗∗*^*p* < 0.01.

**Table 8:** Effect of total glucosides of Xiebai on pathological changes of the thymus on chronic depression model rats.

Group	Number of animals	Dose (mg·kg^−1^)	Number of lymphocytes
Blank group	10	—	527.8 ± 69.0^*∗∗*^
Model group	10	—	440.4 ± 58.0
Fluoxetine hydrochloride group	10	6.6	669.9 ± 83.5^*∗∗*^
High-dose Xiebai total glycosides group	10	200	648.5 ± 75.3^*∗∗*^
Medium-dose Xiebai total glycosides group	10	100	624.1 ± 47.9^*∗∗*^
Low-dose Xiebai total glycosides group	10	50	500.5 ± 34.5^*∗*^

*Note*. Compared with the model group, ^*∗*^*p* < 0.05 and ^*∗∗*^*p* < 0.01.

**Table 9:** Effect of total glucosides of Xiebai on pathological changes of the adrenal gland in rats with chronic depression.

Group	Number of animals	Dose (mg·kg^−1^)	Adrenal cortex thickness
Blank group	10	—	625.7 ± 71.1^*∗∗*^
Model group	10	—	942.9 ± 148.1
Fluoxetine hydrochloride group	10	6.6	728.5 ± 134.2^*∗∗*^
High-dose Xiebai total glycosides group	10	200	726.9 ± 92.3^*∗∗*^
Medium-dose Xiebai total glycosides group	10	100	800.7 ± 153.3^*∗*^
Low-dose Xiebai total glycosides group	10	50	847.5 ± 123.5

*Note*. Compared with the model group, ^*∗*^*p* < 0.05 and ^*∗∗*^*p* < 0.01.

**Table 10:** Effect of total glucosides of Xiebai on pathological changes of the spleen in chronic depression model rats.

Group	Number of animals	Dose (mg·kg^−1^)	Hair growth center diameter
Blank group	10	—	11.1 ± 3.35^*∗∗*^
Model group	10	—	5.1 ± 1.79
Fluoxetine hydrochloride group	10	6.6	12.5 ± 2.22^*∗∗*^
High-dose Xiebai total glycosides group	10	200	12.9 ± 2.13^*∗∗*^
Medium-dose Xiebai total glycosides group	10	100	8.3 ± 1.49^*∗∗*^
Low-dose Xiebai total glycosides group	10	50	7.4 ± 1.17^*∗*^

*Note*. Compared with the model group, ^*∗*^*p* < 0.05 and ^*∗∗*^*p* < 0.01.

## Data Availability

The data used to support the findings of this study are available from the corresponding author upon request.

## References

[1] Yue Li., Wu J., Huang G. (2014). Research status of comorbid metabolic syndrome in depression. *Sichuan Mental Health*.

[2] Zhuang L., Zhan S., Kong Y. (2018). Research progress of traditional Chinese medicine rehabilitation therapy based on hepatic main drainage theory. *Journal of Integrated Traditional and Western Medicine on Cardiovascular and Cerebrovascular Diseases*.

[3] Huang L. (2016). A review of the research on traditional Chinese medicine in the treatment of depression. *Modern Vocational Education*.

[4] Xia W., Qiu W., Fang X. (2018). Based on the theory of “spleen thinking “to observe the expression of brain-derived neurotrophic factor, serotonin, dopamine and norepinephrine in gastroesophageal reflux disease. *Chinese Journal of Integrated Traditional and Western Medicine*.

[5] Wang Z., Li L., Gao L. (2018). Exploring the pathogenesis of Chinese medicine for depression based on the theory of “innate and acquired”. *Research of Traditional Chinese Medicine*.

[6] Yue L., Bai G. (2013). Research status of depression and anxiety disorder. *Medical Review*.

[7] Deng W., Zhang H. (2017). Research status of neuroimmunological related targets in the pathogenesis of depression. *Chinese Journal of Clinical Pharmacology*.

[8] Liu Y., Liu M. (2017). Advances in pharmacology research of Xiebai decoction. *Information on Traditional Chinese Medicine*.

[9] Qiao F., Cai W., Yan Ke. (2016). Research progress of traditional Chinese medicine Xiebai. *World Chinese Medicine*.

[10] Han X., Hu F., Tian F. (2015). Research progress and evaluation of animal models of depression. *Clinical Medicine Practice*.

[11] Chen Y., Tao Li., Sun S. (2017). Effects of Jieyu Anshen Recipe on learning and memory function in chronic mild stress depression animal model. *Chinese Journal of Clinical Pharmacology*.

[12] Cao L., Ming B., Fang X., Wang C., Mingsan M. (2016). Analysis of animal models of depression based on clinical features. *Journal of Neuropharmacology*.

[13] Chen J., Lin X., Liu L. (2018). Protective effect of epigallocatechin gallate on chronic mild unpredictable stress-induced depression mice. *Chinese herbal medicine*.

[14] Surana A. R., Wagh R. D. (2018). Phytochemical analysis and antidepressant activity of ixora coccinea extracts in experimental models of depression in mice. *The Turkish Journal of Pharmaceutical Sciences*.

[15] Xu W., Zhou X. (2016). Research progress on pathogenesis and monotherapy of depressive disorder in traditional Chinese medicine. *Journal of Integrated Traditional and Western Medicine on Cardiovascular and Cerebrovascular Diseases*.

[16] Jiang X., Jin Y., Xiang R. (2017). Research status of traditional Chinese medicine treatment for depression. *Gansu Medical Journal*.

[17] Xu E., Mingsan M., Shang L. (2017). New progress in the treatment of traditional Chinese medicine based on cytokine and neuro-endocrine pathogenesis of depression. *Henan Traditional Chinese Medicine*.

[18] Yang X., Zhang L., Lei S. (2017). Correlation between anxiety, depression and TCM constitution. *Chinese Journal of Integrated Traditional and Western Medicine*.

[19] Jia C., Xu Q., Du Y. (2014). Clinical study on the treatment of post-stroke depression in elderly patients with traditional Chinese medicine qi and activating blood circulation and relieving stagnation method. *Chinese Journal of Traditional Chinese Medicine and Pharmacy*.

[20] Seki K., Yoshida S., Jaiswal M. K. (2018). Molecular mechanism of noradrenaline during the stress-induced major depressive disorder. *Neural Regeneration Research*.

[21] Cheng B., Fang X., Mingsan M. (2014). Molecular mechanism of depression and characteristics of Chinese medicine treatment of depression. *Journal of Traditional Chinese Medicine*.

[22] Zheng Y. P., Wang F. X., Zhao D. Q. (2018). Predictive power of abnormal electroencephalogram for post-cerebral infarction depression. *Neural Regeneration Research*.

[23] Shen P. P., Hou S., Ma D. (2016). Cortical spreading depression-induced preconditioning in the brain. *Neural Regeneration Research*.

[24] Mittal N., Hurn P., Schallert T. (2016). Exploring a need for improved preclinical models of post-stroke depression. *Neural Regeneration Research*.

[25] Wang L., Liu H., Hu H. (2017). Historical changes of Xiebai source plants of traditional Chinese medicine. *China Journal of Traditional Chinese Medicine*.

[26] Sheng H. (2013). Research progress on chemical constituents and pharmacological effects of Xiebai. *Pharmaceutical Research*.

[27] Akbarzadeh G., Daniali H., Javdzadh M., Caes L, Ranjbar S, Habibi M (2018). The relationship of parental pain catastrophizing with parents reports of children’s anxiety, depression, and headache severity. *Iranian Journal of Child Neurology*.

[28] Sun X., Wu H., Zhang P. (2013). Advances in research on chemical constituents and pharmacological activities of Xiebai formulas. *Chinese pharmacy*.

[29] Qian Y., Chang W., He X. (2016). Emotional dysregulation of ADHD in childhood predicts poor early-adulthood outcomes: a prospective follow up study. *Research in Developmental Disabilities*.

[30] Gao W., Qudair Baig A., Ali H., Sajjad W., Reza Farahani M. (2017). Margin based ontology sparse vector learning algorithm and applied in biology science. *Saudi Journal of Biological Sciences*.

[31] Akyol K., Alacacioglu D., Ellidokuz K. (2017). THE effects of adjuvant chemotherapy on serum adma and endothelin-1 levels in early stage breast cancer patients (izmir oncology group (IZOG) study. *Acta Medica Mediterranea*.

[32] Kumar D. (2017). Screening antianxiety and antioxidant profile of stems and leaves of blue variety of clitoria ternatea L. *Indian Journal of Pharmaceutical Sciences*.

[33] Kapusuz Gencer Z., Balbaloğlu Ö., Özkiriş M., Saydam L. (2017). Does fibromyalgia have an effect on hearing loss in women?. *Turkish Journal of Medical Sciences*.

